# Macroeconomic Image Analysis and GDP Prediction Based on the Genetic Algorithm Radial Basis Function Neural Network (RBFNN-GA)

**DOI:** 10.1155/2021/2000159

**Published:** 2021-11-22

**Authors:** Mingxun Zhu, Zhigang Meng

**Affiliations:** ^1^School of Economics and Management, Changsha Normal University, Changsha 410100, China; ^2^School of Computer Engineering and Applied Mathematics, Changsha University, Changsha 410003, Hunan, China

## Abstract

The prediction of gross domestic product (GDP) is a research hotspot, and its importance is self-evident. Its complex internal change mechanism also increases the difficulty of analyzing GDP data. The genetic algorithm (GA) is applied to the parameter design of the radial basis function neural network (RBFNN) based on genetic algorithm optimization (RBFNN-GA). An economic zone GDP image prediction model is proposed, which realizes the optimal design of the center vector, the base width vector of the RBFNN node function, and the weight between the hidden layer and output layer. Based on the GDP data over the years, this paper uses the RBFNN-GA prediction model to analyze and predict the GDP image and compares the image prediction results. The results show that the genetic algorithm is used to optimize RBFNN, which gives full play to the advantages of the two algorithms. The relative error of the RBFNN-GA prediction model is only 3.52%. Compared with the prediction results, the prediction accuracy is significantly higher than the ARIMA time series model and GM (1,1) model.

## 1. Introduction

Gross domestic product (GDP) is not only the most important indicator to measure national economic development but also a comprehensive reflection of economic operation. It is of great significance to analyze and predict the annual, medium-, and long-term GDP and put forward the policy ideas of GDP and economic development. The provincial economy is an important part of the national economy and is relatively independent. Therefore, many research literatures believe that the provincial economy is a relatively independent research object and an important research level of macroeconomics [1, 2]. Although the current economic operation is generally stable, to achieve better and more effective sustainable development in the future, we should constantly summarize the problems exposed on the development road and solve them in time [3]. In recent decades, China's economy has been in a state of rapid development and at the leading level in the world. However, behind the rapid development, it has also paid a heavy price. The original extensive development consumes too many resources, which makes the existing environmental resources bear a high load. In such an economic environment, it is of great significance to predict the future GDP and optimize the industrial structure.

Great progress has also been made in economic image prediction technology at home and abroad. GDP image prediction belongs to the prediction of the economic field. The earliest prediction methods used in the economic field include the time series prediction method, regression analysis prediction method, and econometric method [4, 5]. Because GDP itself is a time series data, this method is widely used. Regression analysis is also often used in economic forecasting. With the rapid development of machine learning and artificial intelligence, the neural network has made great progress in the 1980s. The reason why the neural network can be widely used in the economic field is not only because it has accurate prediction and simple operation but also because it has strong learning ability and can deal with complex nonlinear mapping relations, especially for the nonlinear mapping problems with complex internal structure relations and many influencing factors [6].

In the process of economic image analysis and prediction, most of the models are nonlinear because of the complex influencing factors of the research object. The traditional image analysis and prediction methods have large errors, and the accuracy is difficult to meet the requirements [7]. In this study, the radial basis function neural network (RBFNN-GA) based on the genetic algorithm is used to analyze the economic image and predict the growth law, find out the proportion and role of various economic departments in the economy, and find out the economic differences between cities in the province and the economic development advantages of various regions and the development prospects of various economic sectors under the influence of the new national macroeconomic policies and the world economic situation.

The innovative contribution of this paper is to propose an economic zone GDP image prediction model, which realizes the optimal design of the center vector, base width vector, and the weight of the hidden layer and output layer of the RBFNN node function. Based on the GDP data over the years, the RBFNN-GA prediction model is used to analyze and predict the GDP image, and the image prediction results are compared. The simulation effect of the RBFNN controller designed in this paper is better than the traditional LQR method. Compared with traditional algorithms, the genetic algorithm is used to optimize RBFNN, which gives full play to the advantages of the two algorithms.

## 2. Related Work

In recent years, the emerging artificial intelligence neural network has become the focus of attention of many scholars. Literature [8] uses a computer simulation neural network to study and train data and finally predicts nonlinear data. Because the neural network belongs to the nonlinear system, processing nonlinear data also shows incomparable advantages over the traditional model theory. Literature [9] puts forward a data mining time series pattern algorithm based on fuzzy sets. Literature [10] studies the fractal characteristics of some time series, analyzes the R/S analysis in fractal theory, and uses R/S method to find the change rule from the time series with fractal characteristics to predict the future development trend of the series. Literature [11] proposes a similarity search algorithm based on dynamic time warping technology, which obtains the sequence matching by calculating the shortest warping path between time series data and compares the comprehensive control time series data by clustering analysis based on different distance measures, which greatly improves the calculation accuracy and has strong robustness to amplitude difference, noise and linear drift. Literature [12] uses the neural network to predict multifactor time series data, inputs two pieces of related information in the neural network at the same time, and then uses it to predict; the predicted value is much better than the previous regression analysis results. However, in recent years, the network is mainly used in the prediction of time series analysis and regression analysis. Literature [13] is more accurate than traditional forecasting methods in predicting time series data by multifactor comprehensive analysis of neural networks. Therefore, the neural network has become the focus of domestic scholars for a time. Literature [14] studies the modeling mechanism of neural network, combines a variety of forecasting methods to make time series forecasting, and uses the actual economic data for analysis and calculation. Practice has proved that the accuracy is still higher than the traditional forecasting technology.

Literature [15] first uses K-means clustering algorithm to determine the center of the hidden layer basis function, which is widely used in RBFNN, but the disadvantage of this algorithm is that it is too sensitive to the initial center of clustering. Literature [16] proposes an orthogonal least squares algorithm, which selects the input data that has the greatest influence on the network output as the center of hidden nodes every time and adds the data to RBFNN one by one until a suitable network structure is constructed. Literature [17] constructs RBFNN by taking the support vector as the center of the hidden node. It has been proved that RBFNN based on the support vector has better performance than ordinary RBFNN. Literature [18] proposed an orthogonal least squares algorithm for the RBFNN gene. For learning outliers, a new robust RBFNN is proposed in literature [19], which has a fast learning rate and reasonable network structure, can be used to fit constant value functions and is robust to outliers. Literature [20] puts forward a robust learning algorithm combined with improved the genetic algorithm (GA), which can improve the generalization performance of RBFNN, eliminate noise, and reveal the training data rules, but this algorithm is relatively complex.

Innovative ideas of this paper: in many related literatures of the GDP forecast, we find that the author sometimes only uses one forecast analysis method. A single forecasting method cannot be compared with other forecasting methods, and it is difficult to determine its accuracy. Therefore, in this paper, we use the GA to optimize RBFNN, combined with the grey system theory. By establishing RBFNN-GA, the GDP of Shandong Province is predicted. The RBFNN-GA prediction method can overcome the shortcomings of RBFNN, such as slow learning convergence speed, difficult to ensure convergence to the global minimum point, and difficult to determine the network structure, and greatly improve the precision and accuracy of model prediction.

## 3. Research Method

### 3.1. Basic Theory of the GA and RBFNN

#### 3.1.1. Genetic Algorithm

The GA is an intelligent optimization algorithm in view of the survival of the fittest and genetic laws. The GA first initializes the solution of the problem to get a set of random solutions and regards the random solutions as a population, while the solutions within the population as chromosomes in biology [21]. In the process of evolution, the quality of chromosomes will be good or bad. The GA uses fitness function to evaluate the quality of each chromosome and gets the chance that the independent solution will survive to the next generation. Usually, the higher fitness function value corresponds to the higher probability of chromosome survival. Therefore, the GA then replicates high-quality chromosomes, and after a series of basic operations such as selection, mutation, and mating, a new population is generated and the offspring in this population will be closer to the optimal solution. After generations of reproduction, the evolution does not end until the individuals who meet the quantity of iteration termination or produce the best fitness function value.

The specific steps of GA are shown in Figure 1:

1. Determine the coding strategy: select the appropriate fitness function to determine the range or size of genetic parameters, including population size, operation methods such as selection, crossover and mutation, and crossover and mutation probability.
2. Coding chromosome: usually, binary coding strategy is adopted for coding operation, and the system will randomly generate initialization population.
3. Calculate the individual fitness function value and evaluate the quality of each chromosome.
4. The next generation of the new population is formed by a series of genetic operations, including selection, crossover, and mutation.
5. Judging whether the fitness value meets the target or not, if not, returning to step (3) and continuing to execute the operation flow until the termination confirmation condition is met.

#### 3.1.2. Principle of RBFNN

RBFNN is a three-layer feedforward network with a single hidden layer [22], and the network structure is shown in Figure 2.

Figure 2 shows RBFNN of *l* − *m* − *n* structure. The quantity of nodes in the input layer is *l*, the quantity of nodes in hidden layer is *m*, and the quantity of nodes in output layer is *n*. *x*=[*x*_1_, *x*_2_,…,*x*_*l*_]^*T*^ ∈ *R*^*l*^ is the input vector of the network, *W* ∈ *R*^*m*×*n*^ is the output weight matrix, the output of the network is *y*=[*y*_1_, *y*_2_,…,*y*_*n*_]^*T*^, and Φ_*j*_(*∗*) is the activation function of the *j* th hidden node.

The most notable feature of RBFNN is that the basis function of hidden layer nodes is distance function, that is, RBF is used as the activation function. RBF is radially symmetric about a center point of *n* -dimensional space, and the farther the input is from the center point, the lower the activation degree, which is called the local characteristics of hidden layer nodes. Therefore, each hidden layer node of RBFNN has a data center.

It can be seen from Figure 2 that the *k* th output of RBFNN can be expressed as follows:

(1) $$\begin{array}{c} y_{k}=\sum_{j=1}^{m}w_{j}\Phi_{j}\left(\left\|x-c_{j}\right\|,\sigma_{j}\right), \end{array}$$

where *c*_*j*_ is the center vector of the *j* th hidden node, the dimensions of *x* and *c*_*j*_ are the quantity of nodes in the input layer, and *σ*_*j*_ is the width of the basis function.

It can be seen from the structure of RBFNN that the process of constructing and training RBFNN is to make it determine the quantity of hidden layer neurons, the center and width of each hidden layer basis function, and the output weight, among which the most important one is to resolve the center of basis function. The training process of RBFNN is shown in Figure 3.

There are many forms of RBF, many of which satisfy the Micchelli theorem, and its characteristic is that the quantity of hidden nodes is equal to the quantity of input samples. The following three RBFs satisfy the Micchelli theorem [23, 24].

Gaussian function:

(2) $$\begin{array}{c} \phi \left(r\right)=\exp\left(-\frac{r^{2}}{2\sigma^{2}}\right). \end{array}$$

Multiquadratic function:

(3) $$\begin{array}{c} \phi \left(r\right)=\frac{1}{1+\exp\left(r^{2}/\sigma^{2}\right)}. \end{array}$$

Inverse polyquadratic function:

(4) $$\begin{array}{c} \phi \left(r\right)=\frac{1}{{\left(r^{2}+\sigma^{2}\right)}^{1/2}}. \end{array}$$

### 3.2. GDP Prediction Model of the Shandong Economic Region in China Based on RBFNN Neural Network Improved by the GA

#### 3.2.1. Improved RBFNN Algorithm Based on GA Optimization

The main parameters that need to be adjusted in the training process of RBFNN are the center of the node transfer function of the hidden layer, the variance *σ*, and the connection weights between the hidden layer and output layer, which are obtained by training RBFNN.

At present, several commonly used neural network training methods are the fixed method, gradient descent method, and *K*-means clustering algorithm, and so on. Although the algorithm is simple in design and easy to implement, it also has some defects. As a parallel free rein ferret about the optimization method, the GA has all-out ferret about ability [25]. To improve the prediction accurate of RBFNN, the GA is used to optimize the center *c* and variance *σ* of the transfer function and the connection weight *ω* between the hidden layer and the output layer in the training process of RBFNN prediction model so as to improve the training accuracy and generalization ability of the model.

The basic idea of the GA is to start from the initial population, in the light of the rule of survival of the fittest, and improve the population through continuous reproduction process. The algorithm flowchart of GA combined with RBFNN is shown in Figure 4.

The specific steps of the algorithm are as follows:

(1) Individual coding. Individual coding is an important link in GA design, which is composed of the center *c* of the hidden layer transfer function, variance *σ*, and network connection weight *ω*.
(2) Individual evaluation of algorithm. In the GA, the probability that an individual is inherited to the next generation of individuals is determined by the size of individual fitness, which is the key to measure the advantages and disadvantages of the algorithm [26], and the individual fitness is also the only basis for genetic operation. The fitness function of the *i* -th individual in the population is designed as follows:
  (5) $$\begin{array}{c} f=\frac{1}{\sum_{p=1}^{M}\overset{N}{\underset{j}{\sum }}{\left(y_{ij}^{o}-y_{ij}\right)}^{2}+1}, \end{array}$$
where *M* is the quantity of training samples, *N* is the quantity of output nodes, and *y*_*ij*_^*o*^, *y*_*ij*_ is the expected output and predicted output of the network.
(3) Determine the center of RBF. There are *m* × *l* parameters in the center *c*_*i*_=(*c*_*i*1_, *c*_*i*2_,…, *c*_*il*_),  *i*=1,2,…, *m* of RBF, and *c*_*i*_ can be calculated using the given learning samples, that is, the mean clustering method, which is widely used in pattern recognition. The specific calculation steps are as follows [27]:

(1) Take *m* sample values in learning samples as initial values of *c*_*i*_; Group all learning samples according to the nearest RBF center *c*_*i*_. For each basis function center *c*_*i*_ and all samples *x*_*p*_={*x*_1*p*_, *x*_2*p*_,…, *x*_*lp*_},  *p*=1,2,…, *s*, *x*_*p*_ which satisfies the following formula belongs to the subsample set *α*_*i*_ of *c*_*i*_.
  (6) $$\begin{array}{c} \underset{i}{\min}\left[\sum_{j=1}^{l}{\left(x_{jp}-c_{ij}\right)}^{2}\right]. \end{array}$$
(2) *c*_*i*_ is recalculated and *c*_*ij*_=1/*M*_*i*_∑_*p*∈*α*_*i*__*x*_*jp*_ is taken, where *M*_*i*_ is the quantity of samples in the subsample set *α*_*i*_.
(3) Until the center *c*_*i*_ of the basis function no longer changes, the calculation is stopped to obtain the stable value of the center *c*_*i*_ of the basis function. Otherwise, turn to (2) and 3), recalculate *c*_*ij*_, and cycle the calculation until it is stable.
(4) Determine RBF width. Generally speaking, *e*_*i*_ is taken as the average distance between the center *c*_*i*_ of the basis function and the sample patterns in the subsample set *α*_*i*_:
  (7) $$\begin{array}{c} \sigma_{i}^{2}=\frac{1}{M_{i}}{\sum_{p\in \alpha_{i}}\sum_{j=1}^{l}\left(x_{jp}-c_{ij}\right)}^{2}. \end{array}$$
(5) Determine the connection weight between output neurons and hidden neurons. When *σ*_*i*_ and *c*_*i*_ are determined, the corresponding output can be obtained when the learning sample *x*_*p*_ is given. The weight *ω*_*i*_ is solved by GA method, so the total error *E* of the network is established as the objective function:
  (8) $$\begin{array}{c} E=\sum_{p=1}^{s}E_{p}=\frac{1}{2}{\sum_{p=1}^{s}\sum_{k=1}^{n}\left[{\hat{y}}_{k}\left(x_{p}\right)-y_{k}\left(x_{p}\right)\right]}^{2}, \end{array}$$
in which *s* is the quantity of training samples; ${\hat{y}}_{k}\left(x_{p}\right)$ is the actual output; *y*_*k*_(*x*_*p*_) is the expected output.

When the GA method is used for optimization calculation, the goal is to make the *E* value smaller than the preset maximum permissible error.

#### 3.2.2. Establishment of the GDP Forecasting Model in the Shandong Economic Region

In this paper, six main factors affecting China's GDP (unit: 100 million yuan) are adopted as the structure: total export volume (unit: 100 million dollars), fiscal expenditure (unit: 100 million yuan), total retail consumption (unit: 100 million yuan), actually utilized foreign capital (unit: 100 million dollars), fiscal revenue (unit: 100 million yuan), and fixed assets investment (unit: 100 million yuan) In this paper, the classic three-layer feedforward neural network is used to build GDP prediction model [28–31]. There are six nodes in the input layer, which correspond to the above six structural variables. The quantity of nodes in the hidden layer is usually determined according to empirical formula:

(9) $$\begin{array}{c} s=\sqrt{m+n}+a, \end{array}$$

where *m*, *n* is the quantity of input and output nodes, *s* is the quantity of hidden nodes, and the quantity of hidden nodes in this paper is 5. The quantity of nodes in the output layer is 1, which corresponds to the GDP to be predicted [32].

For the input layer of the neural network, we choose the predicted value of Shandong GDP based on GM(1,1) model. We take the predicted value of Shandong GDP GM(1,1) model from 2010 to 2020 as the input vector of RBFNN-GA, and the actual value of Shandong GDP from 2010 to 2020 as the output vector of RBFNN-GA. The input and output data are normalized, and the neural network model is constructed [33].

Finally, the GA parameters are set. It can be seen from the error change diagram of the model that when GA iterates to 70 generations, the error has become very small, as shown in Figure 5.

Therefore, we set the maximum number of iterations to 70; The population size is set to 60. The crossover probability is set to 0.8. The mutation probability is set to 0.1. According to the set initial values of parameters, coding, population generation, adaptability evaluation and detection, selection, crossover, and mutation are carried out. The RBFNN is trained using the optimal weights and thresholds obtained by GA optimization of neural network, and the predicted values of the model are obtained.

To ensure that there are enough samples and enough differences between samples, the sampling frequency used in this paper is 1 year, and the sample data are GDP data from 2010 to 2020. The specific ideas are as follows:

1. First, learn from 6 sample points from 2010 to 2015, and then use the trained network to predict the GDP value in 2016
2. Advance the training sample points by one, that is, learn from 6 sample points from 2011 to 2016 and then predict the GDP value in 2017
3. And so on, until the GDP in 2020 is predicted

Data processing before neural network learning has a vital impact on the network. The numerical changes of the above six structural variables may be quite different, which cannot be directly used in the training of neural networks; otherwise, the learning speed and accuracy of the networks will be seriously affected.

Data normalization refers to a method which is often used to preprocess the original data before comprehensive processing. Its main function is to normalize the numerical magnitude of each parameter to be studied to the same or basically the same scale so as to avoid that some parameters are highlighted because of their large numerical magnitude and others are suppressed because of their small numerical magnitude in further data processing; otherwise, the result will cause distortion of the processing effect. On the other hand, it makes the preprocessed data show some unique characteristics. Before training, the influence factors of samples are transformed as follows:

(10) $$\begin{array}{c} {\bar{X}}_{j}=\frac{X_{j}-X_{j\min}}{X_{j\max}-X_{j\min}},\;j=1,2,\ldots ,6, \end{array}$$

where *X*_*j*max_ and *X*_*j*min_ represent the maximum value and minimum value of the *j* th influence factor *X*_*j*_ in six groups of training samples, and ${\bar{X}}_{j}$ represents the normalized influence factor value. After the above processing, the values of the six structural variables are all transformed into [0, 1], which is taken as the input value of the network.

## 4. Discussion and Analysis of Results

### 4.1. Simulation Analysis of Algorithm Performance

The inverted pendulum itself is a natural unstable body, which can be stabilized only by effective methods. Therefore, typical control problems such as nonlinearity, system robustness, and tracking can be effectively reflected in the research process of its control. In this section, through the designed RBFNN controller, the double inverted pendulum system is simulated and controlled by Matlab, and the results show the effectiveness of RBFNN-GA.

First, the control effect of the double inverted pendulum is simulated by the simulation module, and the simulation of fixed interference and random interference is carried out by simulating the Simulink module. The application environment is Matlab7.1. The module is selected in the Simulink toolbox of Matlab to build the control loop. Compared with the traditional linear quadratic regulator (LQR) fixed interference model and random interference model, the influence of interference on the control simulation curve is analyzed. Selecting the step function as the input of the system, the simulation results using RBFNN controller and LQR method are shown in Figures 6 and 7.

Comparing Figure 6 with Figure 7, it can be seen that both methods can stabilize the inverted pendulum system, but the overshoot and steady-state error of the double inverted pendulum controlled by the RBFNN controller in the proposed method are smaller than that of the LQR method.

After many comparative tests, it is found that *K* = 4.5 is the optimal working point of the RBFNN controller. At this time, the overshoot, steady-state error, and response time of each variable of inverted pendulum system are reduced, and the controller realizes stable control of the system, as shown in Figure 8.

After the inverted pendulum achieves stable control, the same disturbance force of 0.1 N is applied to the centroid of the trolley. The simulation results of the two control methods are shown in Figures 9 and 10.

Comparing Figure 9 with Figure 10, it can be seen that the two control methods can restore stability after adding the same fixed disturbance of 0.1 N when using the traditional LQR method, the inverted pendulum system will restore its equilibrium state after 4 s, but when using the RBFNN controller, the inverted pendulum will restore its equilibrium state in only about 2 seconds.

### 4.2. Prediction and Analysis of GDP by GA Optimization RBFNN

It is of great significance to analyze, estimate, and infer the trend of GDP, although for so many years, people from all walks of life have been keen on forecasting GDP. Because the data are easy to obtain and comes from the website of the National Bureau of Statistics, it is very accurate and reliable. Judging from China's current policies, the emphasis on GDP may have declined slightly, which makes us think more about the importance of forecasting GDP data.

In this section, we select the GDP data of Shandong Province from 2010 to 2020 and use MATLAB software to forecast the GDP of Shandong Province in 2020 by establishing GA optimized RBFNN, namely RBFNN-GA.

Using the trained network, input the 50th data after logarithm and difference to predict the GDP data in 2020, then input the GDP and fiscal expenditure data from 2010 to 2020 into the trained network, then push the data back, and finally get the simulated and predicted values. After analyzing and predicting the reprocessed data, the predicted values from 2010 to 2020 are compared with the real values as shown in Figure 11.

It can be seen from Figure 11 that the prediction accuracy of neural network is very high, and the fitting value is very close to the real value.

In this section, we will compare and analyze the relative errors of auto regressive integrated moving average (ARIMA) time series, grey model and RBFNN-GA, and the average relative errors of the whole model. The relative error between the actual value and the predicted value of GDP in 2020 and the average error of model fitting are compared and analyzed.  Figure 12 shows the error analysis results of prediction results.

From Figure 12, we can see that the relative error between the predicted value and the actual value of RBFNN-GA 2020 is 3.52%, and the average error of model fitting is 1.36%. Compared with the other two methods, the prediction results of the RBFNN model based on GA optimization are more satisfactory.

By forecasting the GDP of Shandong Province, we can find that the traditional time series model is inferior to the neural network. However, the time series model is a prediction model with a complete set of modeling process and test methods. It has complete theory and simple operation, and it is very applicable on the premise that only short-term data need to be predicted and the prediction accuracy is not high. The grey model established using the grey system theory is also a set of forecasting models with complete modeling process and theoretical basis. It needs a small number of samples and does not need regular distribution. Its operation is simple and easy to operate. Therefore, the grey forecasting model is usually applied to some short-term forecasting.

## 5. Conclusion

In this paper, the predicted value of Shandong GDP GM(1,1) model from 2010 to 2020 is taken as the input vector of RBFNN-GA, and the actual value of Shandong GDP from 2010 to 2020 is taken as the output vector of RBFNN-GA. The input and output data are normalized, and the neural network model is constructed. Through the analysis of RBFNN, this paper proposes to establish the forecasting model of the Shandong economic region GDP based on GA optimization and verifies the optimized forecasting model by simulation. The trained neural network module is modeled by Simulink and simulated, and the fixed interference experiment is carried out on the simulation model. Experimental results show that the simulation effect of RBFNN controller designed in this paper is better than the traditional LQR method. It is proved that the designed RBFNN controller has good robustness and stability. The prediction results show that the predicted value of RBFNN-GA model fits the actual value very well, and the average relative error is only 3.52%. Compared with ARIMA time series model and grey GM(1,1) model, the prediction accuracy is obviously improved. However, the research in this paper is still insufficient in the prediction model data set, and more simulation methods are needed to verify in the future research.

## Figures and Tables

**Figure 1:** GA step.

**Figure 2:** RBFNN structure.

**Figure 3:** RBF training flowchart.

**Figure 4:** Algorithm flowchart of combining GA with RBFNN.

**Figure 5:** Error variation diagram.

**Figure 6:** Simulation curve of RBFNN controlling inverted pendulum.

**Figure 7:** Simulation curve of the LQR control inverted pendulum.

**Figure 8:** Simulation curve of inverted pendulum system under *K* = 4.5.

**Figure 9:** Simulation curve of RBF control for the inverted pendulum.

**Figure 10:** Simulation curve of LQR control of inverted pendulum.

**Figure 11:** The actual value of GDP is fitted with the predicted value of RBFNN-GA.

**Figure 12:** Error analysis of prediction results.

## Data Availability

The data used to support the findings of this study are available from the corresponding author upon request.
